# An Adaptive Learning Image Denoising Algorithm Based on Eigenvalue Extraction and the GAN Model

**DOI:** 10.1155/2022/5792767

**Published:** 2022-02-09

**Authors:** Feng Wang, Zhiming Xu, Weichuan Ni, Jinhuang Chen, Zhihong Pan

**Affiliations:** Guangzhou Xinhua University, Guangzhou, China

## Abstract

This paper proposes a self-adjusting generative confrontation network image denoising algorithm. The algorithm combines noise reduction and the adaptive learning GAN model. First, the algorithm uses image features to preprocess the image and extract the effective information of the image. Then, the edge signal is classified according to the threshold value to suppress the problem of “excessive strangulation,” and then the edge signal of the image is extracted to enhance the effective signal in the high-frequency signal. Finally, the algorithm uses an adaptive learning GAN model to further train the image. Each iteration of the generator network is composed of three stages. And then, we get the best value. Through experiments, it can be seen from the data that the article algorithm is compared with the traditional algorithm and the literature algorithm. Under the same conditions, the algorithm can ensure the operating efficiency while having better fidelity, and it can still denoise at the same time. The edge signal of the image is preserved and has a better visual effect.

## 1. Introduction

The generation of image information will inevitably be more or less accompanied by the generation of noise. Noise is a factor that hinders human sense organs from understanding the received source information. We can define it as an unpredictable, random error. It will have a certain impact on the collection, input, and processing of image information and the final output results. Especially in the process of input, collection, and transmission of image information, if the input is accompanied by large noise, it will definitely have an adverse effect on the subsequent processing process and the processing result. The purpose of denoising is to improve the image and solve the interference problem of the actual image.

With the continuous development of technology, human access to information is obtained through human vision, hearing and touch, and other senses, the vast majority of which information is derived from human vision. And in real life, image acquisition is vulnerable to external interference to form noisy images, and in the process of image segmentation and parameter estimation of noisy images, it will cause errors in the resulting image so that the image denoising processing will become the current research hot spot in the field of image processing [1–5]. In 1992, Donoho proposed the small wave threshold atrophy method; the algorithm with its own denoise superiority quickly attracted people's attention, but its tendency to “overstrangling” wavelet coefficient and cannot optimally represent the line and surface singularity in the image, so that the wavelet transformation in the image denoising has certain limitations [6, 7], but denoising in the past, there is still the problem of fidelity. With the development of artificial intelligence technology, multimodal fusion is an inevitable trend, and multimodal fusion can make more effective use of the characteristics of the image. In practice, a large amount of labeled data is difficult to obtain, but GAN can solve this problem very well [8, 9]. Therefore, the problem of how to combine GAN and noise reduction came into being.

This paper proposes an image denoising algorithm, which is based on a model that generates an adaptive adjustment against the network. It combines noise reduction and the adaptive learning GAN model, preprocesses the image by combining image characteristics, increases the effective information quantity of the image while reducing the amount of image calculation, and then uses the GAN model with adaptive learning to further denoise the image, so as to obtain the best noise removal effect. In order to avoid the phenomenon of “overstrangling” in the process of noise reduction, the referenced threshold classifies its edge signal and then extracts the edge signal of the image to enhance the effective signal in the high-frequency signal while deleting the negligible signal in the image. Each iterative update of the generator network *λ* consists of three stages. In the end, we obtain the key areas in the image and self-learn to obtain the best value for the individual.

## 2. Generative Adversarial Networks

The generative adversarial network (GAN) was proposed by Goodfellow, which uses convolutional neural networks to train image samples [10, 11]. As a probability generation model, the generation against the network has been applied to many visual tasks, especially in the excellent performance of the image generation direction. The network structure is generated as shown in Figure 1.

The purpose is to let the generator generate data similar to the real data distribution to achieve a fake effect. In terms of data prediction, the training generator introduces images into the generation of the neural network and, through training, reduces the difference between the two so that the distributor cannot distinguish the authenticity of the generated data. Since the difference between the generated data distribution *P*_*G*_ and the real data distribution *P*_Data_ cannot be calculated, therefore, the discriminator uses a data sampling method to count the divergence of the two and then distinguish them.

The objective function is

(1) $$\begin{array}{c} V\left(G,D\right)=E_{x∼P_{\text{data}}}\left[\log\;D\left(x\right)\right]+E_{x∼P_{G}}\left[\log\left(1-D\left(x\right)\right)\right]. \end{array}$$

Among them, *E*(∗) is the mathematical expectation value, and *D*(∗) is the result of the differential output. The objective function of maximizing judgment is the dispersion of generated data and real data. According to the distribution dispersion, the prediction function can be obtained:

(2) $$\begin{array}{c} G^{*}=\arg\underset{G}{\min}\underset{D}{\max}V\left(G,D\right). \end{array}$$

GAN can generate generated samples similar to the real data distribution, but there are difficulties in training, data cannot be obtained, difficult to converge, and pattern collapse, and some studies have proposed variations of the GAN to improve the model. When there is no overlap between the generated data and the real data distribution, the dispersion of the two data distributions is constant, Log2, which can lead to the disappearance of gradients and make it difficult for the model to train.

Broadly speaking, generators and judges are not enemies, and they are not confrontational relationships. In fact, they are constantly updating and learning on the basis of each other to achieve each other. During the training process, the goal of generating network *G* is to generate as many real pictures as possible to deceive network *D*. *D* is opposite to *G*, and the goal of *D* is to distinguish between false images generated by *G* and real images as much as possible. The two constitute a dynamic “game process.”

The success of the GAN also benefits from the success of confrontational ideas. The idea of confrontation has been introduced into several fields including machine learning and artificial intelligence. The two behaviors of “game” and “competition” contain the characteristics of confrontation. People combine game theory and machine learning to produce game machine learning.

The advantages and disadvantages of the GAN are as follows: compared with other generative models, GAN has the following four advantages:

- From the actual results, GAN seems to produce better samples than other models.
- Most other frameworks require the generator network to have a certain functional form, for example, the output layer is Gaussian. It is important that all other frameworks require that the generator network be distributed with nonzero quality. The generative confrontation network framework can train any type of generator network and can learn to generate points only on thin manifolds close to the data.
- Any generator network and any discriminator will be useful because they do not need to design a model that follows any type of decomposition.
- There is no need for reasoning during the learning process and no need to use the Markov chain for repeated sampling (inference), thus avoiding difficult approximate calculation problems of probabilities.

Compared with VAE, deep Boltzmann machine, NICE, and real NVE, GAN has no lower limit of change. At the same time, compared with deep Boltzmann machines, GAN does not have tricky partition functions. GAN can be generated all at once through samples, instead of repeatedly applying Markov chain operators.

## 3. The Algorithm of This Article

At present, fuzzy method training using synthetic data cannot effectively distinguish real images. In order to solve this problem, this paper proposes a new method of noise reduction and adaptive learning GAN model, that is, by combining image characteristics to preprocess the image so that the target is clear, then use the GAN model with adaptive learning to further denoise the image, and then get the best noise removal effect.

At present, many researchers have proposed many denoising methods for images. However, some denoising methods will blur the details of the image while denoising the image, making the original clear image blurred and unable to be restored. Some are able to get clear images, but the amount of calculation is too large to meet people's needs. Nowadays, the most common wavelet denoising algorithms are the modulus maximum denoising algorithm, correlation denoising algorithm, and threshold denoising algorithm. Through comparative analysis, it is found that the threshold denoising algorithm is the simplest and has the least amount of calculation in the image processing process, has the characteristics of high flexibility and strong denoising ability, and is the most widely used in practical applications. Therefore, this article chooses to use the threshold denoising algorithm to process the image.

### 3.1. Image Noise Reduction Preprocessing

In a noisy image, the real signal of the image is usually a low-frequency or relatively stable signal, while the noise is generally concentrated in high-frequency signals. Wavelet transform can effectively concentrate energy and concentrate it in the low-frequency region. The Gaussian noise presents a Gaussian distribution, and the main signal is distributed in the high-frequency region. Therefore, the proposed algorithm can quantify the threshold of wavelet coefficients by introducing appropriate thresholds to eliminate noise.

Through the study of noisy images, one can find that, in real life, the low-frequency part of the image signal after wavelet transform is composed of the useful signal of the image, and the image noise often exists in the high-frequency part of the image [12].

  Step 1: wavelet decomposition of the noisy signal: choose the appropriate wavelet and the corresponding decomposition layer.  Figure 2 shows a wavelet decomposition diagram of a noisy image.
  Step 2: perform threshold quantization processing on the high-frequency subbands after wavelet decomposition. Threshold processing of different scales is realized by the threshold, and the corresponding estimated wavelet coefficients are obtained.
  Step 3: reconstruct the obtained signal through your transformation of wavelet coefficients. Finally, the denoised signal is obtained. That is, the wavelet coefficients of the low-frequency subband and other high-frequency subbands are quantized by the threshold, and the signal is reconstructed to obtain the latest estimated signal $\hat{f}\left(t\right)$.

The selection and quantification of the threshold and the classic threshold denoising function are as follows.

Threshold:

(3) $$\begin{array}{c} \lambda =\sigma *\sqrt{2\;\log\;N}. \end{array}$$

By measuring each detail signal, it can be filtered. Among them, *σ* is the standard deviation of the noise, and *N* is the length or scale of the signal. It is defined as follows:

(4) $$\begin{array}{c} {\hat{\omega }}_{i,j}=\left\{\begin{array}{cc} \omega_{i,j}, & \left|\omega_{i,j}\right|>\lambda ,\\ 0, & \left|\omega_{i,j}\right|\leq \lambda . \end{array}\right. \end{array}$$

Finally, the reconstructed data of the image can be obtained.

### 3.2. Noise Reduction (Detail Protection)

Combining the inherent visual characteristics of the human eye, this paper finds that the entropy value of the image can truly reflect the image signal [13–19], but in the actual computer process, the maximum entropy threshold is calculated in a relatively large amount. Therefore, in the process of noise reduction, after the graying of the image, because the image signal is mainly distributed with area 0 and region 1, the probability in regions 2 and 3 is usually set to 0, which greatly simplifies the calculation in the mathematical model.

Research found that, after adaptive decomposition, the edge signals in the high-frequency signal are effectively concentrated [20–28], while the high-frequency signal is mainly used to represent the edge signal of the image, which inevitably shows some noise signals and weak edge signals, if these signals are deleted, it will not affect the overall quality of the image, and how to effectively separate these signals from the edge signal will have a certain impact on the compression of the image.

By analyzing the edge characteristics of its image, we find out the characteristics:

1. Along the gradient direction, the detection is carried out in a certain range, the maximum value is retained, and M_*S*_*f*(*i*, *j*)=1 can be obtained. If the nonmaximum value is deleted, M_*S*_*f*(*i*, *j*)=0 can be obtained.
2. The edge signal is generally a point with a more intense grayscale change, i.e., the corresponding mode value is relatively large, while the corresponding mode value of the noise signal is relatively small.

Therefore, according to the distribution characteristics of the image signal, this paper classifies the image to achieve the compression processing of the image. The method is as follows:

(5) $$\begin{array}{c} W\left(i,j\right)=\left\{\begin{array}{cc} W\left(i,j\right), & M_{s}f\left(i,j\right)>=\lambda ,\\ 0, & M_{s}f\left(i,j\right)<\lambda . \end{array}\right. \end{array}$$

Edge signal function: $M_{s}f\left(x,y\right)=s\sqrt{{\left(\partial F/\partial x\right)}^{2}+{\left(\partial F/\partial y\right)}^{2}}$.

(6) $$\begin{array}{c} F_{s}\left(x,y\right)=\sum_{\left(i,j\right)\in N_{s}\left(x,y\right)}f\left(i,j\right)\phi_{s}\left(x-i,y-j\right),\\ \frac{\partial F_{s}\left(x,y\right)}{\partial x}=\sum_{\left(i,j\right)\in N_{s}\left(x,y\right)}f\left(i,j\right)\frac{\partial }{\partial x}\phi_{s}\left(x-i,y-j\right),\\ \frac{\partial F_{s}\left(x,y\right)}{\partial y}=\sum_{\left(i,j\right)\in N_{s}\left(x,y\right)}f\left(i,j\right)\frac{\partial }{\partial y}\phi_{s}\left(x-i,y-j\right),\\ \frac{\partial }{\partial x}\phi_{s}\left(x-i,y-j\right)={\frac{1}{s^{3}}\frac{\partial \phi \left(u,v\right)}{\partial u}|}_{\left(u,v\right)=\left(x-i/s,y-j/s\right)},\\ \frac{\partial }{\partial y}\phi_{s}\left(x-i,y-j\right)={\frac{1}{s^{3}}\frac{\partial \phi \left(u,v\right)}{\partial v}|}_{\left(u,v\right)=\left(x-i/s,y-j/s\right)}. \end{array}$$

Among them, 0 ≤ *x*, *y* ≤ *N*.

The edge signal in the high-frequency signal is detected, the edge signal is classified by the reference threshold, the edge signal of the image is extracted to enhance the effective signal in the high-frequency signal, and the negligible signal in the image is deleted.

At the same time, in order to avoid excessive denoising, a new threshold is proposed; that is, $\lambda =2^{a}\sigma \sqrt{2\;\log\left(N^{2}\right)}$.

Among them, *a* is the number of filtered stages, *N*^2^ is the maximum scale size of the image signal, and *σ* is the noise standard estimation of the contourlet transform. This paper reduces the appearance of “overstrangling” phenomenon by combining the nature of the image signal and thus improves the accuracy of the denoising algorithm.

According to the inherent characteristics of human vision, the article classifies high-frequency signal information and combines with a new threshold denoising algorithm to effectively remove image noise. Through experiments, the algorithm in this paper can reduce the coding overhead of the denoising algorithm while ensuring the quality of the denoised picture.

By observing Figure 3, it is not difficult to find that this algorithm can effectively remove speckle noise. It can be seen that the processed image has enhanced the contrast of the image, but there are still blurry edges and loss of details.

### 3.3. Adaptive GAN to Improve Image Quality

Image super-resolution, referred to as super-resolution (SR), generally refers to the magnification resolution. For example, if you change the resolution from 256 × 256 to 512 × 512, the magnification scale is 2. Obviously, this is an ill-posed problem of making pixels out of nothing, and there is no unique solution. The image is superdivided, and the application scenarios are naturally wide. The general method is to take the low-resolution (LR) image as the input of the method and process it to obtain the high-resolution (HR) image. Nowadays, quite a lot of papers are self-made LR-HR image pairs as training sets. For example, the LR is obtained by downsampling the original image HR, and then the mapping learning from LR to HR is performed, but when applied to practice, is the relationship between LR and HR a self-righteous “downsampling” relationship? This is probably unknown and difficult to simulate.

Due to the weak correspondence between the random input and pictures, GAN-generated images are prone to misalignment. Also, because the discriminator judges the image as a whole, the generated pictures have stronger continuity and can generate clearer pictures.

When processing images, the pixel loss function similar to the mean square error cannot recover some details that are lost in the downsampling process. Minimizing the mean square error is by finding a reasonable pixel average value, but the processing result of this method is usually too smooth, which will lead to poor perception quality.

The GAN provides a very advanced learning architecture in generating very high-quality natural image research. The architecture of the GAN helps to facilitate the reconstruction of regions that move into the search space. This may contain images that are as real as photos, making the images obtained by the GAN closer to natural images.

Each iteration of the generator network includes three stages [29–31], which enable the generator to quickly and accurately locate the focus area in the image.

(1) *Variation:* Introduce a random noise signal *z*. In the new round of update process using the gradient penalty loss function of this paper, and for the generation of the network gradient penalty loss function is *L*(*G*, *D*) calculated only for noise data, which makes the network according to the parameters updated.
  (7) $$\begin{array}{c} L\left(G,D\right)=E_{z∼P_{z}}\left[D\left(z\right)\right]-E_{z∼P_{z}}\left[D\left(z\right)\right]-\lambda_{\text{gp}}E_{z∼P_{z}}\left[{\left({\left|\left|\nabla_{x}D\left(z\right)\right|\right|}_{2}-1\right)}^{2}\right],\\ L_{\text{MSE}}\left(G,D\right)=L\left(G,D\right)+\lambda_{\text{MSE}}L_{\text{MSE}}\left(G\right). \end{array}$$
Among them, *λ*_gp_ is the weight parameter. *P*_*z*_ is the noise data distribution.
(2) Assess:
In order to learn the correct distribution of training samples and improve the stability of model training, this paper selects an evaluation mechanism that uses the loss function to select the best sample under the screening of the discriminator. The following is the evaluation mechanism:
The quality score of the generated samples and the diversity of the generated samples are the embodiment of the quantification of the adaptive score at this stage: **F**=**F**_**q**_+*γ ***F**_**d**_.
**F**_**q**_ is the quality score, **F**_**d**_ is the diversity score, and *γ* is the ratio parameter of the two. Through the evaluation mechanism, the highest adaptability score is calculated, and the size of the highest score is calculated so that the global optimal score can be obtained. By analogy, until the end of the first generation to the last generation, the optimal value is obtained by comparison, and then the adaptive score is updated.
(3) Select:
According to the evaluation mechanism to select the optimal individual, the other low scores will gradually decay so that the generation network has a certain direction, and choose the optimal value of the individual.

## 4. Experimental Results and Analysis

In order to verify the validity of this method, verify that the algorithm can denoise while retaining image edge information. Since the GAN is a deep learning model, the game between the generation network and the confrontation network is used to improve the results of the generation network. In this paper, PyCharm is used to simulate the algorithm and to compare with the existing traditional algorithm [32] and literature algorithm [33] by processing the same noisy image.

### 4.1. Objective Indicators of Image Denoising

The experimental hardware environment is the processor Intel Corei7-7700, clocked at 3.60 GHz, memory 12 GB, NVIDIA TITAN Xp. The software environment is Windows 10, 64 bit, Python 3.6, and TensorFlow. In order to verify the denoising effect of the proposed algorithm on noisy images, the ImageNet image dataset is selected in the article and combined with the images in real life; 100 × 100, 128 × 128, and 256 × 256 images are selected. Tests were performed at Gaussian noise levels of 10, 20, 30, 40, and 50. On the experimental dataset, when the Gaussian noise standard deviation *σ* of the noise image is larger, the peak signal-to-noise ratio (PSNR) is smaller, and the image distortion is more. On the contrary, the smaller *σ*, the larger the PSNR and the better the denoising effect.

This paper verifies the fidelity effect of the algorithm by comparing the PSNR value of each algorithm.  Table 1 is a comparison data table of the PSNR value obtained by different denoising algorithms through experiments.

It can be seen from Table 1 that, in the case of different noise standard deviations of the same noisy image, by analyzing the PSNR value, it can be seen that the data obtained by the algorithm in this paper are better than the literature algorithm and the traditional algorithm. The data of the algorithm in this paper are compared with those of the traditional algorithm, and the average PSNR value is 10.48 dB higher. Compared with the literature algorithm, the PSNR value of the algorithm in this paper is 6.56 dB higher, which effectively proves the image fidelity capability of the algorithm in this paper.

In order to verify the influence of the noise figure on the algorithm time, this article records the time consumed by the algorithm under the aforementioned environment and draws it into a graph, as shown in Figure 4.

By observing Figure 4, it is not difficult to find that, as the noise figure increases, the time consumed by each algorithm increases. Among them, the curve of the literature algorithm consumes the most, both of which are above the time curve of the traditional algorithm and the article algorithm. The time curve obtained by the algorithm of the article is basically the same as the traditional algorithm.

### 4.2. Iterative Effect Comparison Experiment

This article observes the PSNR value based on the ImageNet dataset and the CIFAR-10 dataset. We analyze the change data of PSNR as the number of iterations increases and express it through a graph.  Figure 5 shows the PSNR curves of three different sizes of images as the number of iterations increases.

It is not difficult to find from the figure that the algorithm in this paper has a better denoising effect in different sizes. After the number of iterations reached 15 K, the growth rate of PSNR also slowed down, and finally, our network results reached a stable value.

### 4.3. Running Time

In order to verify the algorithm, the experiment selects standard image library images and evaluates the average running time of the algorithm based on the same standard. The results are shown in Table 2.

It is not difficult to see from Table 2 that the algorithm in this paper is significantly better than the traditional algorithm in terms of speed. The reason is that although the computational complexity of the literature algorithm code has been significantly reduced after multiple optimizations, the attention-based denoising algorithm needs to extract images for iterative training models to achieve effective denoising, so the computational complexity is relatively high. However, the algorithm in this paper can significantly improve the operating efficiency by simply reducing it for the first time and then scoring and selecting the image. It can be seen from Table 2 that in terms of time, the time of the algorithm in this paper is basically the same as that of the traditional algorithm. These prove the feasibility of the algorithm.

### 4.4. Denoising Effect Comparison Experiment

In order to verify the superiority of the algorithm in the image denoising effect, the pictures of the two actual scenes are selected for simulation experiments, and the denoising effect of each algorithm is shown, where Figures 6 and 7 show the original images.

By observing Figures 8–10, one can see that the image effect processed by the algorithm in this paper is significantly improved compared with the traditional algorithm and the literature algorithm. And the image details and image sharpness processed by the algorithm in this paper are better than the other two algorithms.

The proposed algorithm selects a complex image to perform related operations to verify the algorithm's processing effect on image details.  Figure 7 is a high-altitude shooting with complex content. The effect is shown in the following.

By observing Figures 11–13, one can see that the algorithm in this paper compares the noise reduction simulation of the traditional algorithm and the literature algorithm. It can be seen that the algorithm can denoise the noisy image while still retaining the edge signal of the image and has a good performance. It has better visual effect.

## 5. Conclusion

This paper proposes a self-adjusting generative confrontation network image denoising algorithm. The algorithm includes noise reduction and the adaptive learning GAN model. It preprocesses the image first by combining image characteristics to make the target clear. Then, the algorithm in this paper uses the GAN model with adaptive learning to further denoise the image and then obtains the best denoising effect. The threshold value quoted in the process of noise reduction avoids the phenomenon of “overstrangling” and improves the effective signal in the high-frequency signal. In the GAN model, iterative updates are performed through operations such as mutation, evaluation, and selection. Self-learning of the generator can quickly and accurately locate the key areas in the image to obtain the optimal value. The results show that the proposed algorithm can effectively denoise while retaining the image signal, which is consistent with the expected effect. However, with the explosive growth of the amount of image data, how to optimize the algorithm to improve the efficiency of image denoising execution is a problem that needs further research.

## Figures and Tables

**Figure 1:** A counternetwork structure.

**Figure 2:** Wavelet decomposition diagram of the noisy image.

**Figure 3:** Denoising effect diagram of the GAN.

**Figure 4:** The influence curve of the noise figure on algorithm time.

**Figure 5:** The PSNR curve of three different sizes of images as the number of iterations increases.

**Figure 6:** Original image.

**Figure 7:** Original image.

**Figure 8:** Traditional algorithm.

**Figure 9:** Document algorithm.

**Figure 10:** Article algorithm.

**Figure 11:** Traditional algorithm.

**Figure 12:** Document algorithm.

**Figure 13:** Article algorithm.

**Table 1:** The PSNR value data table for the results obtained by different denoising algorithms.

*σ*	PSNR (dB)			
	Noisy images	Traditional denoise	Literature algorithms	Article algorithm
10	24.21	29.32	35.95	37.05
20	21.34	29.12	31.02	38.21
30	18.91	25.15	30.12	39.34
40	16.32	30.57	32.58	37.12
50	14.22	26.11	30.22	40.97

**Table 2:** Average running time of different algorithms.

Algorithm	Panda (s)	Duck (s)	Cliff (s)	Average running time (s)
Traditional algorithm	0.823	0.992	0.859	0.891333
Document algorithm	1.467	1.036	1.904	1.469
Article algorithm	0.993	0.838	0.882	0.904333

## Data Availability

The data used to support the findings of this study are available from the corresponding author upon request.
